# Acupuncture-Moxibustion Combined with Rehabilitation Training Is Conducive to Improving the Curative Effect, Cognitive Function, and Daily Activities of Patients with Cerebral Infarction

**DOI:** 10.1155/2022/4430345

**Published:** 2022-05-21

**Authors:** Ding Zhang, Liemi Huang, Lun Zhang, Xinghua Gui, Jiping Tao, Pengli Zeng, Min Ding

**Affiliations:** ^1^Department of Rehabilitation Medicine, Wuhan Sixth Hospital, Affiliated Hospital of Jianghan University, Wuhan, 430000 Hubei Province, China; ^2^Department of Urology, Wuhan Sixth Hospital, Affiliated Hospital of Jianghan University, Wuhan, 430000 Hubei Province, China

## Abstract

**Objective:**

To elucidate the effect of acupuncture-moxibustion combined with rehabilitation training (RHT) on the curative effect, cognitive function (CF), and activities of daily living (ADL) of patients with cerebral infarction (CI).

**Methods:**

This study enrolled 150 patients with CI admitted to the Wuhan Sixth Hospital, Affiliated Hospital of Jianghan University from June 2020 to July 2021. Among them, 80 patients who were treated with acupuncture-moxibustion combined with RHT were included in the research group, and 70 patients who received acupuncture-moxibustion alone were included in the control group. The efficacy, CF, and ADL were observed in both groups, and the influences of the two therapies on serum uric acid (UA), high-sensitivity C-reactive protein (hs-CRP), and cystatin C (Cys-C) were compared. Among the various indexes, the CF of patients was assessed by the Montreal Cognitive Assessment (MoCA), and the ADL was evaluated by the Barthel index.

**Results:**

After treatment, the research group presented significantly better efficacy, CF, and ADL than the control group, with lower levels of serum UA, hs-CRP, and Cys-C than the control group and before treatment.

**Conclusion:**

Acupuncture-moxibustion combined with RHT can inhibit serum UA, hs-CRP, and Cys-C levels of patients with CI while improving the curative effect, CF, and ADL, which is worthy of clinical promotion.

## 1. Introduction

Cerebrovascular diseases are acute neurological disorders and common systemic diseases, which are common killer diseases of human beings due to high mortality, disability, and recurrence rates [1]. Cerebral infarction (CI) is the most common type of cerebrovascular disease, with the main clinical pathogenic factors including cerebral thrombosis, lacunar infarction, and cerebral embolism [2]. According to epidemiological data, the number of patients with CI has reached 33 million worldwide and may increase to 77 million by 2030 [3]. The pathogenesis of CI is related to the imbalance of cerebral blood supply leading to ischemic necrosis or encephalomalacia, which further causes neuron damage and brain dysfunction [4]. Patients with CI will suffer varying degrees of damage to their cognitive function (CF) and activities of daily living (ADL) due to the development of the disease, which will impose heavy economic and psychological burden to patients and their families [5]. Previous studies have shown that CI can lead to severe sequelae and even disability and death if optimal clinical decisions are not made promptly [6]. Therefore, designing a more effective and reliable treatment scheme for CI is of great significance for reducing the high mortality, disability, and recurrence rates of the disease.

Acupuncture-moxibustion is a traditional Chinese treatment technique that uses sterile metal needles to stimulate specific acupoints, so as to activate the body's self-healing process and halt disease progression [7]. Acupuncture-moxibustion has been extensively applied to the treatment of angina pectoris, myocardial infarction, CI, and other hypoxic-ischemic diseases [8–10]. Its therapeutic effect in CI may be to enhance neuroplasticity by inhibiting post-ischemic inflammatory response while stimulating neurogenesis and angiogenesis [11]. A large number of animal experiments have confirmed that acupuncture-moxibustion has a neuroprotective effect in CI, which is realized through biological processes such as increasing cerebral blood flow, modulating oxidative stress, inhibiting glutamic acid excitotoxicity, maintaining blood-brain barrier integrity, and reducing apoptosis [12]. Rehabilitation training (RHT) is a targeted training method aimed at alleviating post-CI cognitive dysfunction, which can improve the brain function of patients with cognitive dysfunction after CI from multiple dimensions such as attention, memory, communication ability, and executive capacity [13]. Wang et al. [14] also proposed that RHT combined with acupuncture-moxibustion can significantly enhance the curative effect of patients with CI-induced hemiplegia, with a high safety.

This paper mainly discusses the effects of acupuncture-moxibustion combined with RHT on the curative effect, CF, and ADL of CI patients, aiming at providing new approaches for the treatment of CI.

## 2. Materials and Methods

### 2.1. General Data

In this retrospective study, 150 patients with CI admitted to the Wuhan Sixth Hospital, Affiliated Hospital of Jianghan University from June 2020 to July 2021 were selected. Of them, 80 cases treated with acupuncture-moxibustion combined with RHT were set as the research group, and the rest 70 patients treated by acupuncture-moxibustion alone were set as the control group. This study was approved by the Ethics Committee of hospital, and all the subjects provided informed consent.

### 2.2. Inclusion and Exclusion Criteria

Inclusion criteria: treatment-naive patients with confirmed diagnosis of CI; the National Institutes of Health Stroke Scale (NIHSS) score ≥ 1 point [15]; no previous history of craniocerebral trauma, cerebrovascular events, or encephalitis.

Exclusion criteria: cerebral hemorrhage, brain trauma, or brain tumor; other malignant tumor(s); poor treatment compliance; severe organ or systemic diseases; pregnant or lactating patients.

### 2.3. Treatment Methods

Patients in the control group were treated with acupuncture-moxibustion therapy. Baihui, Fengchi, Fengfu, Touwei, and philtrum-philtra were used as the main acupoints. For those with hemiplegia, Quchi, Neiguan, Hegu, Huantiao, Weizhong, and Sanyinjiao were additionally selected. Scalp-acupuncture: after routine disinfection, 0.25 mm × 40 mm fine needles were used for three-phase head acupuncture, and the needle tip was inserted at a 15° angle to the scalp. The needle was twirled quickly for 2 min once every 10 min, with the needle twirling speed of 200 times/min, for a total of 3 times. Then, the needle was retained for 30 min. Body-acupuncture: local disinfection was first carried out, followed by acupuncture using 0.30 mm × 40 mm fine needles. After needling response, the needle was inserted using the lifting-thrusting method and then twirled for 3 min with the needle twirling speed of 60 times/min. The needle was then retained for 30 min. The acupuncture-moxibustion therapy was performed once daily for 5 times per week, for a total of 4 weeks.

On the basis of the above treatment, the research group was supplemented with RHT that was conducted 60 min every day, 5 times a week, lasting for 4 weeks. The training contents are as follows:

1. Attention was assessed through gaze training and Schulte Grid Puzzle. Before the training, red dots were drawn on the blackboard from top to bottom and from big to small. Patients were asked to stare at the red dots sequentially and extended the blinking time as much as possible. In the case of eyestrain, they were allowed to take a short rest. Before Schulte grid training, 1-25 digits were filled in randomly in 25 squares, and patients were asked to finger read in sequence at the fastest speed
2. *Intensive Memory Training*. A certain number of numbers, pictures, and words were used for patients to remember repeatedly and were recalled 5 seconds later. Patients were then asked to say what they saw. The training was repeated several times, and the difficulty was increased according to the memory training effect
3. Daily life-related topics, such as age estimation and item evaluation, were formulated according to the education level of patients
4. ADL and communication-related training, such as sorting and arrangement of articles, were carried out
5. *Orientation Training*. Patients were asked to identify seasons, rooms, addresses, friends, relatives, and nurses to form concepts of time, space, and characters
6. *Balance Training*. Nursing staff guided patients to perform bedside standing and sitting balance exercises to exercise their balance ability, so as to help them perform rotation activities and forward and backward movements under the correct standing and sitting posture
7. *Sports Training*. Nursing staff instructed patients to walk or go up and down stairs appropriately, while paying attention to ensuring patient safety
8. *Skill Training*. Patients were instructed to perform vertebral body exercises, wiping the table, basketball control, etc., to exercise their hand and upper limb functions

### 2.4. Efficacy Evaluation

The treatment efficacy was assessed according to the degree of NIHSS score reduction [16]. Cured was indicated if the patient could completely take care of himself/herself, with a reduction of NIHSS score ≥ 91%. If the patient could basically take care of himself/herself, with a NIHSS score reduced by 46-90%, it was considered as markedly effective; if the score reduction was between 18% and 45%, and the patient could partially take care of himself/herself, it was considered effective; ineffective referred to a score reduction of <18% and the inability to take care of himself/herself.

### 2.5. Outcome Measures

1. *Efficacy*. The patients were evaluated for efficacy, and the overall response rate was the percentage of the sum of cured, markedly effective and effective cases in the total number of patients
2. *CF*. The CF of patients was evaluated based on the Montreal Cognitive Assessment (MoCA) scale [17], with a score of 0-30. The score is directly proportional to the CF of patients
3. *ADL*. The Barthel index [18], with a score of 0-100, was used to analyze the ADL of patients. The higher the score, the better the ADL
4. *Serum Indices*. Fasting cubital venous blood (5 mL) was sampled from patients and centrifuged (4°C, 1500×g) for 15 min to obtain the serum. Serum levels of uric acid (UA), highly sensitive C-reactive protein (hs-CRP), and cystatin C (Cys-C) were detected by enzyme-linked immunosorbent assay (ELISA) [19] strictly following the instructions of corresponding human ELISA kits (Shanghai Fantai Biotechnology Co., Ltd., Cat. Nos. FT-P32112R, FT-P31428R, FT-P31384R)

### 2.6. Statistical Analysis

Data analysis and image rendering were performed by SPSS 17.0 (IBM Corp., Armonk, NY, United States) and GraphPad Prism 6 (GraphPad Software, Inc., San Diego, CA, USA), respectively. Counting data were represented by number of cases/percentages (*n*/%), and the difference between groups was identified by the Chi-square test. Measurement data were expressed as Mean ± SD; independent samples *t*-test was used to compare data between groups, and paired *t*-test was used for intragroup comparisons before and after treatment. The significance level was set at *P* < 0.05. Of note, ∗ indicates *P* < 0.05 in this study, while ∗∗ indicates *P* < 0.01, a level with more statistical significance than *P* < 0.05.

## 3. Results

### 3.1. Baseline Data

The research group and the control group were comparable in age, average age, sex, onset time, hypertension, coronary heart disease, hyperlipidemia, diabetes, family history of CI, and marital status, with no statistical significance (*P* > 0.05) Table 1.

### 3.2. Effect of Acupuncture-Moxibustion Combined with RHT on Curative Effects of CI Patients

The overall response rate was 74.29% in the control group and 87.50% in the research group, with statistical significance between the two groups (*P* < 0.05) Table 2.

### 3.3. Effect of Acupuncture-Moxibustion Combined with RHT on CF of CI Patients

The MoCA score, which showed no significant difference between the two groups before therapy (*P* > 0.05), increased significantly in both groups after treatment (*P* < 0.01); and there was a significant difference between the two groups after treatment (*P* < 0.01) Figure 1.

### 3.4. Effect of Acupuncture-Moxibustion Combined with RHT on ADL of CI Patients

The ADL of patients was compared using the Barthel index. The data revealed no statistical difference in the Barthel index between groups before treatment (*P* > 0.05). After treatment, the Barthel index score elevated significantly in both groups (*P* < 0.01), with a more significant increase in the research group compared with the control group (*P* < 0.01) Figure 2.

### 3.5. Effect of Acupuncture-Moxibustion Combined with RHT on Serum UA, hs-CRP, and Cys-C Levels in Patients with CI

Serum UA, hs-CRP, and Cys-C levels, which presented no significant difference between the two groups before therapy (*P* > 0.05), decreased statistically after treatment (*P* < 0.01), with more significant reductions in the three indexes in the research group compared with the control group (*P* < 0.01) Figure 3.

## 4. Discussion

CI is a major threat to human health, which can lead to brain injury, disability, and even death worldwide [20]. The principle of TCM treatment of CI is to promote blood circulation and remove stasis, while acupuncture-moxibustion can not only improve blood circulation but also relieve muscle spasm of patients and enhance limb mobility [21, 22]. At present, more and more researchers use acupuncture-moxibustion combined with RHT as a therapeutic strategy for poststroke spastic paralysis, hip fracture, cerebral palsy, and other diseases, which can improve the clinical efficacy, ADL, and CF of patients to varying degrees [23–25]. This study mainly analyzes the clinical effect of acupuncture-moxibustion combined with RHT for the treatment of CI, hoping to provide a new choice for the management of CI.

We included 80 CI patients (research group) who were treated with acupuncture-moxibustion combined with RHT and 70 CI patients (control group) treated with acupuncture-moxibustion alone. Acupoints such as Baihui, Fengchi, and Fengfu were selected for acupuncture-moxibustion treatment, as well as Quchi and Neiguan on the affected limb of the patient. Of them, Baihui is related to the function of the brain network system among hippocampus, parietal lobe, and frontal lobe; and stimulating this acupoint is conducive to repairing the neurons of patients [26]. Fengchi can improve the blood supply to the brain, while both Fengfu and Baihui are on the Du channel and can be used as acupoints for the treatment of brain diseases [27, 28]. In addition, Quchi can stimulate circulation, and Neiguan can improve brain energy metabolism and blood oxygen supply [29]. In this study, it was found that the total effective rate of patients treated with acupuncture-moxibustion combined with RHT was significantly higher compared with those treated with acupuncture-moxibustion alone (87.50% vs. 74.29%). This may be related to the fact that patients also received RHT in addition to acupuncture-moxibustion therapy, which trained and activated brain function in many aspects such as attention, memory, communication ability, and executive capacity. We then evaluated patients' CF by the MoCA. The results showed that the MoCA score in the research group was statistically higher than that in the control group and before treatment, suggesting that acupuncture-moxibustion combined with RHT was more conducive to improving the CF of patients. In terms of ADL, the Barthel index of the research group increased significantly after treatment and was higher than that of the control group, which indicated that acupuncture-moxibustion combined with RHT had more prominent advantages in improving patients' ADL. Hu et al. [30] also pointed out that acupuncture-moxibustion combined with RHT more significantly improved the ADL of patients than acupuncture-moxibustion alone, which was similar to the results of this study. Finally, the combination therapy was found to more effectively inhibit serum UA, hs-CRP, and Cys-C levels than acupuncture-moxibustion alone. Serum UA, hs-CRP, and Cys-C are risk factors of cognitive impairment in patients with CI, and the higher their levels, the greater the risk of cognitive impairment [31]. Our research results demonstrate that patients treated with acupuncture-moxibustion combined with RHT have a relatively lower risk of cognitive impairment aggravation.

The novelty of this study is that we evaluated the effectiveness of acupuncture-moxibustion combined with RHT in the treatment of CI from the perspectives of efficacy, CF, ADL, and serum factors and obtained the following results: while improving the curative effect, CF, and ADL of CI patients, acupuncture-moxibustion combined with RHT can inhibit serum UA, hs-CRP, and Cys-C levels. However, this study still has some room for improvement. First, the observation of long-term efficacy can be increased to determine the effect of acupuncture-moxibustion combined with RHT on the long-term efficacy of patients with CI. Second, basic animal research can be conducted to unlock the protective mechanism of acupuncture-moxibustion combined with RHT for patients with CI. Third, increasing the clinical sample size will also play an important role in improving the accuracy of the experimental results. The research will be further improved from the above aspects in the future.

## 5. Conclusion

In summary, acupuncture-moxibustion combined with RHT has a definite positive effect on CI, which can significantly improve the CF and ADL of patients and inhibit the progression of disease by inhibiting serum UA, hs-CRP, and Cys-C levels. Our research provides new clinical reference and insights for the treatment of patients with CI.

## Figures and Tables

**Figure 1:** Effect of acupuncture combined with rehabilitation training on cognitive function of patients with cerebral infarction. Note: research group (*n* = 80), control group (*n* = 70); ∗∗*P* < 0.01.

**Figure 2:** Effect of acupuncture combined with rehabilitation training on activities of daily living of patients with cerebral infarction. Note: research group (*n* = 80), control group (*n* = 70); ∗∗*P* < 0.01.

**Figure 3:** Effect of acupuncture combined with rehabilitation training on serum UA, hs-CRP, and Cys-C levels in patients with cerebral infarction. (a) Comparison of UA between the research group (*n* = 80) and the control group (*n* = 70). (b) Comparison of hs-CRP between the research group (*n* = 80) and the control group (*n* = 70). (c) Comparison of Cys-C between the research group (*n* = 80) and the control group (*n* = 70). Note: ∗∗*P* < 0.01.

**Table 1:** Baseline data of two groups of patients (*n*(%), mean ± SD).

Variables	*n*	Control group (*n* = 70)	Research group (*n* = 80)	*χ* ^2^/*t*	*P*
Age (years)				3.399	0.065
<60	89	36 (51.43)	53 (66.25)		
≥60	61	34 (48.57)	27 (33.75)		
Average age (years)	150	59.29 ± 12.51	60.09 ± 11.07	0.417	0.678
Gender				0.048	0.826
Male	85	39 (55.71)	46 (57.50)		
Female	65	31 (44.29)	34 (42.50)		
Course of disease (d)	150	63.04 ± 32.90	63.99 ± 31.82	0.179	0.859
Hypertension				0.472	0.492
No	62	31 (44.29)	31 (38.75)		
Yes	88	39 (55.71)	49 (61.25)		
Coronary heart disease				1.648	0.199
No	98	42 (60.00)	56 (70.00)		
Yes	52	28 (40.00)	24 (30.00)		
Hyperlipoidemia				2.041	0.153
No	105	45 (64.29)	60 (75.00)		
Yes	45	25 (35.71)	20 (25.00)		
Diabetes mellitus				0.111	0.739
No	127	60 (85.71)	67 (83.75)		
Yes	23	10 (14.29)	13 (16.25)		
Family history of cerebral infarction				3.189	0.074
No	105	44 (62.86)	61 (76.25)		
Yes	45	26 (37.14)	19 (23.75)		
Marital status				0.021	0.884
Single	42	20 (28.57)	22 (27.50)		
Married	108	50 (71.43)	58 (72.50)		

**Table 2:** Efficacy of two groups of patients (*n*(%)).

Groups	*n*	Cured	Markedly effective	Effective	Ineffective	Total effective rate (%)
Control group	70	10 (14.29)	25 (35.71)	17 (24.29)	18 (25.71)	52 (74.29)
Research group	80	16 (20.00)	40 (50.00)	14 (17.50)	10 (12.50)	70 (87.50)
*χ* ^2^ value	—	—	—	—	—	4.294
*P* value	—	—	—	—	—	0.038

## Data Availability

The labeled dataset used to support the findings of this study is available from the corresponding author upon request.
